The article "An Efficient Deep Learning Approach to Pneumonia Classification in Healthcare" was published in 2019. Journal: J Healthc Eng.

# An Efficient Deep Learning Approach to Pneumonia Classification in Healthcare

**DOI:** 10.1155/2019/4180949

**Published:** 2019-03-27

**Authors:** Okeke Stephen, Mangal Sain, Uchenna Joseph Maduh, Do-Un Jeong

**Affiliations:** ^1^Department of Computer Engineering, Dongseo University, Busan, Republic of Korea; ^2^Division of Computer Engineering, Dongseo University, Busan, Republic of Korea; ^3^Department of Civil Engineering, Yeungnam University, Gyeongsan, Republic of Korea

## Abstract

This study proposes a convolutional neural network model trained from scratch to classify and detect the presence of pneumonia from a collection of chest X-ray image samples. Unlike other methods that rely solely on transfer learning approaches or traditional handcrafted techniques to achieve a remarkable classification performance, we constructed a convolutional neural network model from scratch to extract features from a given chest X-ray image and classify it to determine if a person is infected with pneumonia. This model could help mitigate the reliability and interpretability challenges often faced when dealing with medical imagery. Unlike other deep learning classification tasks with sufficient image repository, it is difficult to obtain a large amount of pneumonia dataset for this classification task; therefore, we deployed several data augmentation algorithms to improve the validation and classification accuracy of the CNN model and achieved remarkable validation accuracy.

## 1. Introduction

The risk of pneumonia is immense for many, especially in developing nations where billions face energy poverty and rely on polluting forms of energy. The WHO estimates that over 4 million premature deaths occur annually from household air pollution-related diseases including pneumonia [1]. Over 150 million people get infected with pneumonia on an annual basis especially children under 5 years old [2]. In such regions, the problem can be further aggravated due to the dearth of medical resources and personnel. For example, in Africa's 57 nations, a gap of 2.3 million doctors and nurses exists [3, 4]. For these populations, accurate and fast diagnosis means everything. It can guarantee timely access to treatment and save much needed time and money for those already experiencing poverty.

Deep neural network models have conventionally been designed, and experiments were performed upon them by human experts in a continuing trial-and-error method. This process demands enormous time, know-how, and resources. To overcome this problem, a novel but simple model is introduced to automatically perform optimal classification tasks with deep neural network architecture. The neural network architecture was specifically designed for pneumonia image classification tasks. The proposed technique is based on the convolutional neural network algorithm, utilizing a set of neurons to convolve on a given image and extract relevant features from them. Demonstration of the efficacy of the proposed method with the minimization of the computational cost as the focal point was conducted and compared with the exiting state-of-the-art pneumonia classification networks.

In recent times, CNN-motivated deep learning algorithms have become the standard choice for medical image classifications although the state-of-the-art CNN-based classification techniques pose similar fixated network architectures of the trial-and-error system which have been their designing principle. U-Net [5], SegNet [6], and CardiacNet [7] are some of the prominent architectures for medical image examination. To design these models, specialists often have a large number of choices to make design decisions, and intuition significantly guides manual search process. Models like evolutionary-based algorithms [8] and reinforcement learning (RL) [9] have been introduced to locate optimum network hyperparameters during training. However, these techniques are computationally expensive, gulping a ton of processing power. As an alternative, our study proposes a conceptually simple yet efficient network model to handle the pneumonia classification problem as shown in Figures 1 and 2.

CNNs have an edge over DNNs by possessing a visual processing scheme that is equivalent to that of humans and extremely optimized structure for handling images and 2D and 3D shapes, as well as ability to extract abstract 2D features through learning. The max-pooling layer of the convolutional neural network is effective in variant shape absorptions and comprises sparse connections in conjunction with tied weights. When compared with fully connected (FC) networks of equivalent size, CNNs have a considerably smaller amount of parameters. Most importantly, gradient-based learning algorithms are employed in training CNNs and they are less prone to diminishing gradient problem. Since the gradient-based algorithm is responsible for training the whole network in order to directly diminish an error criterion, highly optimized weights can be produced by CNNs.

## 2. Related Works

Latest improvements in deep learning models and the availability of huge datasets have assisted algorithms to outperform medical personnel in numerous medical imaging tasks such as skin cancer classification [11], hemorrhage identification [12], arrhythmia detection [13], and diabetic retinopathy detection [14]. Automated diagnoses enabled by chest radiographs have received growing interests. These algorithms are increasingly being used for conducting lung nodule detection [15] and pulmonary tuberculosis classification [16]. The performance of several convolutional models on diverse abnormalities relying on the publicly available OpenI dataset [17] found that the same deep convolutional network architecture does not perform well across all abnormalities [18], ensemble models significantly improved classification accuracy when compared with single model, and finally, deep learning method improved accuracy when compared to rule-based methods.

Statistical dependency between labels [19] was studied to arrive at more precise predictions, thereby outperforming other techniques on given 13 images selected from 14 classes [20]. Algorithms for mining and predicting labels emanating from radiology images as well as reports have been studied [21–23], but the image labels were generally constrained to disease tags, thus lacking contextual information. Detection of diseases from X-ray images was examined in [24–26], classifications on image views from chest X-ray were carried out in [27], and body parts segmentation from chest X-ray images and computed tomography was performed in [23, 28]. Conversely, learning image features from text and creating image descriptions relative to what a human would describe are yet to be exploited.

## 3. Materials and Methods

We present the detailed experiments and evaluation steps undertaken to test the effectiveness of the proposed model. Our experiments were based on a chest X-ray image dataset proposed in [29]. We deployed Keras open-source deep learning framework with tensorflow backend [10] to build and train the convolutional neural network model. All experiments were run on a standard PC with an Nvidia GeForce GTX TITAN Xp GPU card of 12 GB, cuDNN v7.0 library, and CUDA Toolkit 9.0.

### 3.1. Dataset

The original dataset [25] consists of three main folders (i.e., training, testing, and validation folders) and two subfolders containing pneumonia (P) and normal (N) chest X-ray images, respectively. A total of 5,856 X-ray images of anterior-posterior chests were carefully chosen from retrospective pediatric patients between 1 and 5 years old. The entire chest X-ray imaging was conducted as part of patients' routine medical care. To balance the proportion of data assigned to the training and validation set, the original data category was modified. We rearranged the entire data into training and validation set only. A total of 3,722 images were allocated to the training set and 2,134 images were assigned to the validation set to improve validation accuracy.

### 3.2. Preprocessing and Augmentation

We employed several data augmentation methods to artificially increase the size and quality of the dataset. This process helps in solving overfitting problems and enhances the model's generalization ability during training. The settings deployed in image augmentation are shown below in Table 1.

The rescale operation represents image reduction or magnification during the augmentation process. The rotation range denotes the range in which the images were randomly rotated during training, i.e., 40 degrees. Width shift is the horizontal translation of the images by 0.2 percent, and height shift is the vertical translation of the images by 0.2 percent. In addition, a shear range of 0.2 percent clips the image angles in a counterclockwise direction. The zoom range randomly zooms the images to the ratio of 0.2 percent, and finally, the images were flipped horizontally.

### 3.3. Model

Figure 3 shows the overall architecture of the proposed CNN model which consists of two major parts: the feature extractors and a classifier (sigmoid activation function). Each layer in the feature extraction layer takes its immediate preceding layer's output as input, and its output is passed as an input to the succeeding layers. The proposed architecture in Figure 3 consists of the convolution, max-pooling, and classification layers combined together. The feature extractors comprise conv3 × 3, 32; conv3 × 3, 64; conv3 × 3, 128; conv3 × 3, 128, max-pooling layer of size 2 × 2, and a RELU activator between them. The output of the convolution and max-pooling operations are assembled into 2D planes called feature maps, and we obtained 198 × 198 × 32, 97 × 97 × 62, 46 × 64× 128, and 21 × 21 × 128 sizes of feature maps, respectively, for the convolution operations and 99 × 99 × 32, 48 × 48 × 64, 23 × 23 × 128, and 10 × 10 × 128 sizes of feature maps from the pooling operations, respectively, with an input of image of size 200 × 200 × 3 as shown in Table 2. It is worthy to note that each plane of a layer in the network was obtained by combining one or more planes of previous layers.

The classifier is placed at the far end of the proposed convolutional neural network (CNN) model. It is simply an artificial neural network (ANN) often referred to as a dense layer. This classifier requires individual features (vectors) to perform computations like any other classifier. Therefore, the output of the feature extractor (CNN part) is converted into a 1D feature vector for the classifiers. This process is known as flattening where the output of the convolution operation is flattened to generate one lengthy feature vector for the dense layer to utilize in its final classification process. The classification layer contains a flattened layer, a dropout of size 0.5, two dense layers of size 512 and 1, respectively, a RELU between the two dense layers and a sigmoid activation function that performs the classification tasks.

## 4. Results

To evaluate and validate the effectiveness of the proposed approach, we conducted the experiments 10 times each for three hours, respectively. Parameter and hyperparameters were heavily turned to increase the performance of the model. Different results were obtained, but this study reports only the most valid.

As explained above, methods such as data augmentation, learning rate variation, and annealing were deployed to assist in fitting the small dataset into deep convolutional neural network architecture. This was in order to obtain substantial results as shown in Figure 4. The final results obtained are training loss = 0.1288, training accuracy = 0.9531, validation loss: 0.1835, and validation accuracy of 0.9373.

CNN frameworks always require images of fixed sizes during training. Thus, to demonstrate the validation performance of our model on variant input data, we reshaped the X-ray images into 100 × 100 × 3, 150 × 150 × 3, 200 × 200 × 3, 250 × 250 × 3, and 300 × 300 × 3 sizes, respectively, trained them three hours each, and obtained their overall average performance as shown in Figure 4 and Table 3.

The larger the size of the transformed images, the lesser the validation accuracy obtained. In contrast, smaller-sized training images induced a slight improvement in validation accuracy as shown in Figure 5. However, the little slips in the validation accuracy do not register substantial impact on the overall classification performance of the proposed model. Larger images also required more training time and computation cost, and the performances of 150 × 150 × 3 and 200 × 200 × 3 image sizes were similar, as shown in Table 3 and Figure 5, respectively. Finally, we propose the 200 × 200 × 3 model since it produced better validation accuracy of approximately 94 percent with a minimal training loss of 0.1835.

## 5. Discussion

We developed a model to detect and classify pneumonia from chest X-ray images taken from frontal views at high validation accuracy. The algorithm begins by transforming chest X-ray images into sizes smaller than the original. The next step involves the identification and classification of images by the convolutional neural network framework, which extracts features from the images and classifies them. Due to the effectiveness of the trained CNN model for identifying pneumonia from chest X-ray images, the validation accuracy of our model was significantly higher when compared with other approaches. To affirm the performance of the model, we repeated the training process of the model several times, each time obtaining the same results. To validate the performance of the trained model on different chest X-ray image sizes, we varied the sizes of the training and validation dataset and still obtained relatively similar results. This will go a long way in improving the health of at-risk children in energy-poor environments. The study was limited by depth of data. With increased access to data and training of the model with radiological data from patients and nonpatients in different parts of the world, significant improvements can be made.

## 6. Conclusions

We have demonstrated how to classify positive and negative pneumonia data from a collection of X-ray images. We build our model from scratch, which separates it from other methods that rely heavily on transfer learning approach. In the future, this work will be extended to detect and classify X-ray images consisting of lung cancer and pneumonia. Distinguishing X-ray images that contain lung cancer and pneumonia has been a big issue in recent times, and our next approach will tackle this problem.

## Figures and Tables

**Figure 1:** Sample images without pneumonia.

**Figure 2:** Sample images with pneumonia [10].

**Figure 3:** The proposed architecture.

**Figure 4:** Performance of the classification model on 200 × 200 × 3 data size.

**Figure 5:** Performance of the classification model on varied data sizes.

**Table 1:** Settings for the image augmentation.

Method	Setting
Rescale	1/255
Rotation range	40
Width shift	0.2
Height shift	0.2
Shear range	0.2
Zoom range	0.2
Horizontal flip	True

**Table 2:** The output of the proposed network architecture.

Layer (type)	Output shape	Turtles
conv2d_9 (conv2D)	(None, 198, 198, 32)	896
max_Pooling2d_9 (MaxPooling2)	(None, 99, 99, 32)	0
conv2d_10 (conv2D)	(None, 97, 97, 64)	18496
max_Pooling2d_10 (MaxPooling2)	(None, 48, 48, 64)	0
conv2d_11 (conv2D)	(None, 46, 46, 128)	73856
max_Pooling2d_11 (MaxPooling2)	(None, 23, 23, 128)	0
conv2d_12 (conv2D)	(None, 21, 21, 128)	147584
max_Pooling2d_12 (MaxPooling2)	(None, 10, 10, 128)	0
flatten_3 (Flatten)	(None, 12800)	0
dropout_3 (Dropout)	(None, 12800)	0
dense_5 (Dense)	(None, 512)	6554112
dense_6 (Dense)	(None, 1)	513

**Table 3:** Performance of the classification model on different data sizes.

Data size	Training accuracy	Validation accuracy
100	0.9375	0.9226
150	0.9422	0.9343
**200**	**0.9531**	**0.9373**
250	0.9513	0.9297
300	0.9566	0.9267
Average	0.94814	0.93012

## Data Availability

The data used to support the findings of this study are included within the article.
